The article "Implementation of Whale Optimization for Budding Healthiness of Fishes with Preprocessing Approach" was published in 2022. Journal: J Healthc Eng.

# Implementation of Whale Optimization for Budding Healthiness of Fishes with Preprocessing Approach

**DOI:** 10.1155/2022/2345600

**Published:** 2022-02-02

**Authors:** Pravin R. Kshirsagar, Hariprasath Manaoharan, Vineet Tirth, Saiful Islam, Sandeep Srivastava, Varsha Sahni, M. Thangamani, M. M. Khanapurkar, Venkatesa Prabhu Sundramurthy

**Affiliations:** ^1^Department of Artificial Intelligence, G.H. Raisoni College of Engineering, Nagpur, India; ^2^Department of Electronics and Communication Engineering, Audisankara College of Engineering and Technology, Gudur, Andhra Pradesh, India; ^3^Mechanical Engineering Department, College of Engineering, King Khalid University, Abha 61411, Asir, Saudi Arabia; ^4^Civil Engineering Department, College of Engineering, King Khalid University, Abha 61411, Asir, Saudi Arabia; ^5^MCA Department, GL BAJAJ Institute of Technology & Management, Greater Noida, India; ^6^Department of Computer Science and Engineering, CT Group of Institute (CTIEMT), Shahpur, I.K.Gujral Punjab Technical University, Jalandhar, Pin 144603, India; ^7^Department of Information Technology, Kongu Engineering College, Perundurai, Tamilnadu, India; ^8^G.H. Raisoni College of Engineering, Nagpur, India; ^9^Center of Excellence for Bioprocess and Biotechnology, Department of Chemical Engineering, College of Biological and Chemical Engineering, Addis Ababa Science and Technology University, Addis Ababa, Ethiopia

## Abstract

This article examines distinctive techniques for monitoring the condition of fishes in underwater and also provides tranquil procedures after catching the fishes. Once the fishes are hooked, two different techniques that are explicitly designed for smoking and drying are implemented for saving the time of fish suppliers. Existing methods do not focus on the optimization algorithms for solving this issue. When considering the optimization problem, the solution is adequate for any number of inputs at time *t*. For this combined new flanged technique, a precise system model has been designed and incorporated with a set of rules using contention protocols. In addition, the designed system is also instigated with a whale optimization algorithm that is having sufficient capability to test the different parameters of assimilated sensing devices using different sensors. Further to test the effectiveness of the proposed method, an online monitoring system has been presented that can monitor and in turn provides the consequences using a simulation model for better understanding. Moreover, after examining the simulation results under three different scenarios, it has been observed that the proposed method provides an enhancement in real-time monitoring systems for an average of 78%.

The article "Implementation of Whale Optimization for Budding Healthiness of Fishes with Preprocessing Approach" was published in 2022. Journal: J Healthc Eng.

## 1. Literature: A Brief Review

For applying the proposed indication on monitoring fisheries with smoking and cutting methods, many existing methodologies have been analyzed, and they are discussed in this section. Since many accurate predictions are needed under water, a smart quality sensor has been designed with a new adaptive system model [1]. The major exertion has concentrated on analyzing the varying nature of fishes, and an ice storage system has been used for storage where only a limited number of measurements have been provided. Consequently, association between index quality and standard quality is provided by selecting a sequencing method that validates calibration and corroboration of sensors. Also, wireless sensors have been integrated, and their performance on water quality has been checked in the western region of Andhra Pradesh where direct field visits have been made for designing an autonomous mode of operation [2]. The researchers examined and created an autonomous vehicle that is capable of traveling inside water and reports corresponding information to the base station. This type of system has been inspected in India for the first time, and it is significantly supportive for all aqua farmers to lead a better quality of life. A review has been prepared by comparing different methods for monitoring the health parameters of each fish [3] that are present inside the water. This type of review provides complete information on the usage of low-power devices that requires only minimum water for improving the productivity in farms. Moreover, the impact of freshwater has also been discussed, but only a small area has been considered, and it is not enough to make a prudent decision since the area of monitoring is much important for aquaculture research.

Moreover, an analytical method for monitoring water quality has been examined [4] under four different categories that even include the existence and nonexistence of different contaminants. For monitoring both physical and biological contaminants, a high-end network setup is needed with low-cost sensors. The major reason for using high-quality setup is to avoid microbes that affect the aqua farms, but the cost of implementation is higher when a high-end network setup is established. Once the fishes are gathered, they should be desiccated for a period of time; therefore, a smoking machine is established [5], which observes only a small quantity of water. However, the setup consists of a closed-loop circulation with Arduino Uno sustenance where high-cost pipes and chambers are established. This method serves as a basic perception of desiccating the fishes within three hours, and it can even be changed from one place to another. Even during the smog period, the fishes can be dehydrated for six hours, but the amount of energy that is consumed for this process is much higher due to the existence of a huge chamber. Therefore, to overcome the drawback of the big-sized chamber that cannot be used in the indoor environment, a machine learning algorithm for smoking fishes has been created [6]. This procedure uses the concept of k-nearest neighbor for receiving the data from the chamber with help of low-cost sensors. But, in most methods, only a binary value is not sufficient to determine the simplicity of prediction. The researchers have also rationalized the old technique of image classification to the video detection method [7] where an automated detection scale has been presented with different time scales. One additional advantage of the aforementioned method is that it paves way for transferring the video to all cable telescopes. But a high number of video nodes is needed for underwater, and it will be difficult to integrate all information from several nodes.

The article "Implementation of Whale Optimization for Budding Healthiness of Fishes with Preprocessing Approach" was published in 2022. Journal: J Healthc Eng.

In a fish processing survey, it is observed that most of the fishes are smoked and expurgated before reaching the final stage [8] that is not good for health. Therefore, it is necessary to monitor the amount of proteins that are present in each fish, and they should be extracted for use in other sources. Furthermore, the researchers have explored that the amount of freshness in fish fillets should also be monitored [9] that is significantly useful for improving the accuracy of the entire system. This procedure can be implemented with multiple ethereal that can store fishes for a period of 12 days, and the high amount of power will be consumed during this process when images are extracted. For both assessment and data processing techniques the components of machine vision applications are extracted [10] that include the size and volume of fishes to be smoked. This type of machine vision application serves as an important component for the automatic processing of aqua food processing techniques. Moreover, for measuring both quality and quantity of fishes, an electronic sensor device has been implemented that detects tongue and nose for electronic authentication process [11]. This type of high advancement needs metal-oxide-semiconductor field-effect transistor electrochemical sensors to be implemented at a high cost.

Additionally, control guidance by the food processing industry for storing vulnerabilities has been provided [12] that serve as a contrivance for all countries to follow highly defined standards in aqua farms. By following these standards, an investigation has been made in the Mediterranean Sea [13] where attrition is prevented and fishes are protected in prematured stage itself. Since most of the process is implemented with sensors, a new system model is necessary; therefore, a semiconductor sensor model has been created [14], and it is integrated with machine vision algorithms. Besides, this system an agent-based simulator has also been introduced in the current system process that provides an inherent mechanism for monitoring fishes [15]. This type of model is having many hidden layers, and all these layers are fulfilled only using the cost of communication channels.

The article "Implementation of Whale Optimization for Budding Healthiness of Fishes with Preprocessing Approach" was published in 2022. Journal: J Healthc Eng.

To improve the health of fishes in underwater, whale optimization algorithm is used. In this study, the behavior of fishes and their presented environment, that is, underwater, are analyzed for the number of sensors deployed. Both environment and fish-related information are analyzed using the sensors. Based on the current state, the performance of optimization is achieved using the sensors.

The rest of this paper is organized as follows.  Section 2 summarizes the precise design methodology in which the proposed system overview is detailed.  Section 4 discusses the proposed optimization algorithm for using the fishers improvement analysis.  Section 5 discusses the results and discussion for the proposed methodology in which the overall results of the designed methodology are highlighted in detail, and finally, the system is concluded with the conclusions and further enhancements.

## 2. Precise Design Methodology

For designing a precise methodology, it is much important to calibrate the sensors, and all the decompositions that are used for smoking fishes must run in a parallel manner. Since parallel operations are performed, a likelihood model has to be formed that performs different sensor operations when data is distributed individually. Therefore, the likelihood function can be established using the following equation:

(1) $$\begin{array}{c} f\left(i\right)=\overset{n}{\underset{i=1}{\sum }}\frac{{\left(\mu_{i}-p_{i}\right)}^{2}}{\sigma_{i}^{2}}, \end{array}$$

where *p*_*i*_ denotes the prediction of sensors for distributed data. *μ*_*i*_ and *σ*_*i*_ represents the mean and variance of given likelihood functions.

Equation (1) denotes that variation in size of fishes with different sizes in the smoking process has been considered using mean and variance functions. Also, during the cutting process, it is difficult to cut the fishes of the same size; therefore, for proper examination of length and breadth, data are predicted using a contact distance sensor that is indicated as LVDT has been integrated inside the corresponding cutting machines. After unknown likelihood values are known in the next step, all measurement counts gained during the cutting process have to be calculated using the following equation:

(2) $$\begin{array}{c} \frac{\text{d}c_{i}}{\text{d}t_{i}}=\mu_{i}\left(1-10^{m_{i}\left(t\right)}\right), \end{array}$$

where *m*_*i*_(*t*) denotes various concentrations in the population of fishes at time *t* = *0* inside the smoking chamber. Equation (2) indicates that all concentrated population values will be segregated with respect to time, and it will be multiplied with mean values that are obtained from equation (1). One major reason for considering all segregated values in terms of time is that each fish will be kept inside the chamber at different times, and for each time, a separate size cannot be given as input likelihood values. Therefore, for cutting the fishes in equal size, it is necessary to separate fishes of different sizes, and all can be kept inside the chamber by following different time periods. In addition, for taking all measurements, it is obligatory to observe that output voltage of sensors during the temperature setting process. Thus, the output voltage in terms of time can be represented as follows:

(3) $$\begin{array}{c} \max\;{\text{volt}}_{i}=\sum_{i=1}^{n}\frac{298K\times e^{{\text{temp}}_{i}\left(1/t_{1}-1/t_{0}\right)}}{e^{{\text{temp}}_{i}\left(1/t_{1}-1/t_{0}\right)}\times g_{i}}, \end{array}$$

where 298*K* represents the initial temperature when fishes are kept inside the chamber for the smoking process. temp_*i*_ denotes distinguishing temperatures between 1,000K and 3,000K. *t*_1_ and *t*_0_ signify different timing characteristics when fishes are smoked inside the chamber. *g*_*i*_ represents greater resistance that is provided when corresponding voltages are divided.

The article "Implementation of Whale Optimization for Budding Healthiness of Fishes with Preprocessing Approach" was published in 2022. Journal: J Healthc Eng.

Equations (1)–(3) indicates that the prediction of sensors should be a variable process and it should be eminent using a statistical test that follows a chi-square distribution as indicated in the following equation:

(4) $$\begin{array}{c} S_{i}^{2}=\sum_{i=1}^{n}\frac{\left(E_{i}-P_{i}\right)}{P_{i}^{2}}, \end{array}$$

where *S*_*i*_^2^ denotes the corresponding sampling times. *E*_*i*_ and *P*_*i*_ represent the observed and predicted values from LVDT sensors, respectively.

In order to establish the relationship between input and output variables, it is necessary to integrate a polynomial regression that is nonlinear in nature as given in the following equation:

(5) $$\begin{array}{c} \theta_{i}=\sum_{i=1}^{n}\gamma_{i}\tau_{i}, \end{array}$$

where *γ*_*i*_ denotes the scaled cutting factor of fishes. *τ*_*i*_ represents the enduring measurement values of LVDT sensors.

If equation (5) is established correctly, then it indicates that the efficiency of the entire process is going to be decided using inclinations of the water quality process where high velocity needs to be applied for smoking fishes by integrating wide channels. Also, it is necessary to find the activity of each fish that is present inside the pond using two different parameters since cutting and smoking methods are used.

(6) $$\begin{array}{c} a_{i}=\sum_{i=1}^{n}e^{\omega_{i}*\vartheta_{i}}, \end{array}$$

where *ω*_*i*_ represents the average swimming time of different fishes inside the pond. *ϑ*_*i*_ denotes the swimming speed of each fish.

Equation (6) is specified to calculate the speed and time of spinning for each fish since it is necessary to differentiate different types of fishes that are present inside the pond. Once the activities of different fishes are known, then the total area of the tarn will be monitored, and the rapidity of the airstream will be converted using control rule as follows:

(7) $$\begin{array}{c} R{\left(i\right)}_{100\text{ m}}={ℵ}_{25}+\frac{E_{i25\text{ m}}}{E_{i14.4\text{ m}}}, \end{array}$$

where *ℵ*_25_ represents the rapidity of the air stream at an altitude of 25 meters. *E*_*i*25 m_ and *E*_*i*14.4 m_ represent the rapidity of the air stream at an altitude of 25 meters and 14.4 meters, respectively.

Equation (7) indicates the control rule where sensors are placed at an altitude of two different meters such as 25 meters and 14.4 meters. After establishing the altitude of each pond, measurement and regulation of the feed process for each fish have to be calculated; this is designed using the following equation:

(8) $$\begin{array}{c} {\text{feed}}_{i}=1-\left(i_{\max}-i_{\min}\right), \end{array}$$

where *i*_max_ and *i*_min_ denotes the maximum and minimum intestine values of each fish, respectively.

Equation (8) denotes that difference between the maximum and minimum intestine values will provide the amount and regulation of feed using calcium-sensing receptors. The perception behind this calculation is to determine the amount of water that is absorbed by each fish in its intestine. In addition, the sensitivity of absorbed water will be measured at various luminescence levels that are exposed by calcium receptors.

## 3. Optimization Algorithm

In this section, an optimization process is introduced for integrating the system model for defined objective functions such as monitoring of pond, measurement, and regulation of feed with proper natural contaminant proportions. Therefore, in the first step, a set of rules have been defined using contention protocols since the load of measurement is higher. For making this contention protocol work, the main node will be divided into many subnodes that is termed as adaptive tree method. The protocol is designed to distribute the work allocated to each sensor node and to provide a collision-free technique, while packets are distributed to intended recipients. With the use of collision-free protocols, collisions do not occur, and the CSMA/CD and CSMA/CA use the possibility of the collisions for the transmission channel that is acquired using any station. Therefore, for every successful packet transmission, an optimal path will be selected, and it can be given statistically as follows:

(9) $$\begin{array}{c} {\text{Prob}}_{i}=\sum_{i=1}^{n}\left[\frac{z_{i}-1}{z_{i}}\right], \end{array}$$

where *z*_*i*_ represents a number of stations struggling to get channel access from the central node.

The article "Implementation of Whale Optimization for Budding Healthiness of Fishes with Preprocessing Approach" was published in 2022. Journal: J Healthc Eng.

Suppose if a station is connected to the corresponding channel in the specified first slot, then the probability rate can be given as follows:

(10) $$\begin{array}{c} z_{i}{\text{prob}}_{i}{\left(1-{\text{prob}}_{i}\right)}^{z_{i}-1}. \end{array}$$

Since many subnodes are present in the media access control sublayer for monitoring the condition of fishes that are present in underwater, the expected number of uniformly distributed stations must be discovered. This is expressed using the following:

(11) $$\begin{array}{c} U_{i}=\;\log_{2}z_{i}. \end{array}$$

For monitoring the entire pond, which is present in underwater using wireless sensors, four different steps are followed in every transmission cycle. In the first phase of transmission, a request for sending data will be sent, and in the next phase, once the request is accepted, entire data will be discarded in current node, and it will be sent back to the requested nodes. In the third and fourth phase data, acknowledgment will be sent from each subnet node that is connected in a pipe-like structure. Moreover, contention-free protocols will use the concept of time-division multiple access where each and every node will be allotted a separate slot for data transmission. At the final stage, all packets will be combined for providing suboptimal congestions, and it can be expressed using the following condition:

(12) $$\begin{array}{c} T_{i,j}=\sum_{i=1}^{n}{\text{Prop}}_{i}+{\text{Prop}}_{j}+T_{i0}+T_{j0}, \end{array}$$

where Prop_*i*_ and Prop_*j*_ denote the propagation delay in seconds. *T*_*i*0_ and *T*_*j*0_ represents the delay from first *i*^th^ and *j*^th^ nodes, respectively.

Whenever protocols are defined using wireless sensors, a large computational complexity will be present that can be solved by the application of the corresponding algorithm. Therefore, in the proposed method, a whale optimization algorithm [16, 17] will be incorporated for optimizing the schedules in control and data transmission phases. The major advantage of selecting a whale optimization algorithm is that it provides an accurate system for allocating different resources in underwater that are consumed by fishes. In addition, the implemented algorithm is having the ability to provide solutions using very few parameters, and even global solutions can be obtained within less period of time. Since the problem is linear, it is necessary to calculate capacity constraints as follows:

(13) $$\begin{array}{c} \sum_{i,j=1}^{n}TW_{ij}\geq AW_{ij}, \end{array}$$

where *TW*_*ij*_ denotes total water supply resource from *i*^th^ to *j*^th^ node. *AW*_*ij*_ represents available water supply resource from *i*^th^ to *j*^th^ node.

The article "Implementation of Whale Optimization for Budding Healthiness of Fishes with Preprocessing Approach" was published in 2022. Journal: J Healthc Eng.

Equation (13) denotes that the total water supply should be greater than or at least equal to the available water supply in different resources. To calculate the current precise solution, distance between whale and generated prey should be observed. This can be calculated using the following equation:

(14) $$\begin{array}{c} \Delta_{i}=\left|d_{w}\left(t\right)-d_{p}\left(t\right)\right|, \end{array}$$

where *d*_*w*_(*t*) and *d*_*p*_(*t*) represent the distance of whale and prey with respect to time.

Subsequently, it is necessary to explore the solution in whale optimization algorithm using exploration phase where two different coefficient will be used for performing a global search that can be expressed using the following equation:

(15) $$\begin{array}{c} d\left(t+1\right)=\bar{d_{t}}-i.j. \end{array}$$

Here *i*, *j* represent two different coefficient that are used in the exploration phase.

Consequently, the aforementioned protocol and algorithm have to be implemented with a system model with different objectives. Therefore, step-by-step implementation is elucidated in Figure 1.

## 4. Results and Discussion

In this section, validation of the system model after integrating whale optimization algorithm by defining a set of rules has been deliberated. Since the proposed method is deciphering multiple objectives, the following three major scenarios are considered:

- Scenario 1: surveillance of tarn
- Scenario 2: regulation of feed
- Scenario 3: proportion of natural contaminant

For these aforementioned scenarios, simulation analysis is performed by incorporating the corresponding hardware setup with Node-RED, and the reproduction is performed offline using MATLAB for better indulgence of day-to-day activities of fishes in underwater.

### 4.1. Scenario 1

In this scenario, the basic parameter that is necessary for monitoring the fish pond is investigated. Since more number of fishes is present in underwater, there is a necessity for monitoring the turbidity level of water inside the tarn. In the proposed exploration, fishes that are present inside the pond are monitored for a period of 20 days uninterruptedly, and all observed data have been stored in the online monitoring system. The data have been imported using MATLAB, and simulation results for scenario 1 have been reflected in Figure 2. If the turbidity level of water is reduced, then fishes can stay inside the water for a long period of time, and hence, level of health can also be increased.

The article "Implementation of Whale Optimization for Budding Healthiness of Fishes with Preprocessing Approach" was published in 2022. Journal: J Healthc Eng.

From Figure 2, it can be observed that for every time period, the maximum and accurate turbidity levels are monitored. Also, if an intelligent sensing device is present, it is possible to evaluate the precise value of turbidity level; therefore, in Figure 2, time period of sensors is reserved for one alignment, and turbidity values that are measured in NBT are reticent for another alignment. After examining the simulated results, it is ascertained that the proposed method using an intelligent sensing device performs well when compared to the existing method. For example, if the time period of sensors is 15,000 minutes, then the level of turbidity for an existing method is 168 NBT, but the proposed method provides the exact turbidity level that is observed as 108 NBT. This proves that within the selected time period and even if the time period is poignant, the proposed method can provide exact turbidity values without any error.

### 4.2. Scenario 2

After examining the turbidity level, the amount of feed that is supplied to fishes must be counteracted; this is examined in this scenario. If the amount of feed is much higher than the body length of fishes, then they cannot move to the exact position, and if it moves inside high depth, then it is difficult for fishermen to catch fishes.

Therefore, this method has been monitored using an intelligent sensing device, and simulation results for determining the amount of feed has been provided in Figure 3. Figure 3 is plotted by considering the body length of fishes that are measured in meters. By measuring the body length of fishes, the amount of feed that is supplied for each fish should be either increased or decreased. From Figure 3, it can be observed that only sensors can monitor the amount of feed in a precise way as compared to the existing method in absence of the intelligent sensing device. For example, if the body length of fish is 13.5 meters, then the amount of feed that needs to be supplied for a day is 10, but in existing methods, only 9 times the fishes are nourished. This will affect the health, and furthermore, it will decrease the lifetime of fishes. Since the proposed method can regulate the correct amount of feed, it can be preferred for real-time monitoring in underwater.

The article "Implementation of Whale Optimization for Budding Healthiness of Fishes with Preprocessing Approach" was published in 2022. Journal: J Healthc Eng.

### 4.3. Scenario 3

This scenario examines the third major parameter that defines the maximum natural contaminant that is present in underwater. In real-time application of fisheries, natural contaminant should be much lesser for preventing the fishes before it enters the red zone region. Therefore, careful experimentation has been processed by establishing sensors, and the percentage of natural contaminant that is mixed with undesirable content has been observed. To realize the percentage of mixture simulation results using observed values are plotted in Figure 4.

Figure 4 is plotted by considering the temperature that is present in underwater where it is varied between 85° and 105°. The major reason for considering the temperature is that for each period of time, the level of contaminants will vary, and if the temperature is much higher, then the original contaminant level will be further reduced.

The growth of fishes will be much higher only when it is present in the bottom layer of water, and if natural contaminants are reduced, fishes will come up to the top level, and in early stages, they will be hooked. Therefore, to avoid this, the proposed method provides the exact amount of natural contaminants that are present in the pond. In this scenario, the proposed method performs much better than the existing method in terms of percentage identification of contaminants and prevents the fishes before it enters the upper layer.

## 5. Conclusions

A new flanged real-time monitoring and examination of fishes in underwater have been introduced with the simulation model in this article. Even though many methods are available for monitoring the state of fishes that are present in underwater, it is necessary that remote checks should be performed using intelligent monitoring devices. Therefore, the major advantage of the proposed method is that it reduces the time of fish vendors as they can able to smoke and dry the fishes within a short period of time. Since this new technique combines monitoring the health of fishes with cutting and smoking techniques a set of rules has been designed with contention protocols since large data is processed. This technique is also integrated with Node-RED for storing central data where users can able to access it using an authentication key. Subsequently, this online monitoring system can provide day-to-day results, and they are integrated with simulation fragments that are executed using MATLAB. It has been experiential that the integrated whale optimization algorithm that is integrated with system model can provide improved results around 78% that is much higher than existing methods. In future, the proposed method can be protracted by introducing robotic technology to further reduce the export time of vendors.

The article "Implementation of Whale Optimization for Budding Healthiness of Fishes with Preprocessing Approach" was published in 2022. Journal: J Healthc Eng.

## Figures and Tables

**Figure 1:** Implementation of WOA for monitoring activities of fishes.

**Figure 2:** Turbidity level of the fish pond.

**Figure 3:** Level of regulating fish feed.

**Figure 4:** Percentage of contaminants in underwater.

## Data Availability

The data sets used and/or analyzed during the current study are available from the corresponding author upon reasonable request.

## References

[1] García M. R., Cabo M. L., Herrera J. R., Ramilo-Fernández G., Alonso A. A., Balsa-Canto E. (2017). Smart sensor to predict retail fresh fish quality under ice storage. *Journal of Food Engineering*.

[2] Shareef Z., Reddy S. R. N. (2018). Wireless sensor network for aquaculture: review, survey, and case study of aquaculture practices in western Godavari region. *Journal of Ambient Intelligence and Smart Environments*.

[3] Akhter F., Siddiquei H. R., Alahi M. E. E., Mukhopadhyay S. C. (2021). Recent advancement of the sensors for monitoring the water quality parameters in smart fisheries farming. *Computers*.

[4] Su X., Sutarlie L., Loh X. J. (2020). Sensors, biosensors, and analytical technologies for aquaculture water quality. *Research: Ideas for Today’s Investors*.

[5] Jayanti T. A. D., Sudarmanto A., Faqih M. I. (2020). Cold smoking equipment design of smoked fish products with closed circulation using temperature and concentration monitoring system based on Arduino Uno. *IOP Conference Series: Materials Science and Engineering*.

[6] Cho J. H. (2020). Detection of smoking in indoor environment using machine learning. *Applied Sciences*.

[7] Marini S., Fanelli E., Sbragaglia V., Azzurro E., Del Rio Fernandez J., Aguzzi J. (2018). Tracking fish abundance by underwater image recognition. *Scientific Reports*.

[8] Ghaly A. E., Ramakrishnan V. V., Brooks M. S., Budge S. M., Dave D. (2013). Fish processing wastes as a potential source of proteins, amino acids and oils: a critical review. *Journal of Microbial & Biochemical Technology*.

[9] Khoshnoudi-Nia S., Moosavi-Nasab M. (2019). Prediction of various freshness indicators in fish fillets by one multispectral imaging system. *Scientific Reports*.

[10] Gümüş B., Balaban M. Ö, Ünlüsayin M. (2011). Machine vision applications to aquatic foods: a review. *Turkish Journal of Fish AquatScience*.

[11] Zaukuu J. L. Z., Bazar G., Gillay Z., Kovacs Z. (2019). Emerging trends of advanced sensor based instruments for meat, poultry and fish quality- a review. *Critical Reviews in Food Science and Nutrition*.

The article "Implementation of Whale Optimization for Budding Healthiness of Fishes with Preprocessing Approach" was published in 2022. Journal: J Healthc Eng.

[12] FDA (2020). *Fish and fishery products hazards and controls guidance*.

[13] Sendra S., Parra L., Lloret J., Jiménez J. M. (2015). Oceanographic multisensor buoy based on low cost sensors for posidonia meadows monitoring in mediterranean sea. *Journal of Sensors*.

[14] Seto S., Kawabe H., Shi L., Shimomura Y., Oyabu T., Katsube T. (2006). Mathematical model of semiconductor gas sensor. *Sensors and Materials*.

[15] García-Magariño I., Lacuesta R., Lloret J. (2017). Abs-Fishcount: an Agent-Based simulator of underwater sensors for measuring the amount of fish. *Sensors*.

[16] Yan Z., Wang S., Liu B., Li X. (2018). Application of whale optimization algorithm in optimal allocation of water resources. *E3S Web of Conferences*.

[17] Mirjalili S., Lewis A. (2016). The whale optimization algorithm. *Advances in Engineering Software*.

